The article "Research on the sustainable design strategies of vernacular architecture in Southwest Hubei—A case study of the First Granary of Xuan’en County" was published in 2024. Journal: PLoS One.

# Research on the sustainable design strategies of vernacular architecture in Southwest Hubei—A case study of the First Granary of Xuan’en County

**DOI:** 10.1371/journal.pone.0316518

**Published:** 2024-12-31

**Authors:** Wei Xu, Qinyu Wang, Hao Deng, Zhenhua Zhu

**Affiliations:** 1 School of Civil Engineering and Architecture, Wuhan Institute of Technology, Wuhan, China; 2 Village Culture and Human Settlements Research Center, Wuhan Institute of Technology, Wuhan, China; 3 Zhengzhou Branch, Henan Communication Construction Management Consulting Co, Ltd, Zhengzhou, China; Central Queensland University, AUSTRALIA

## Abstract

Vernacular architecture, optimized over centuries to create comfortable thermal environments using sustainable design strategies and local materials, can offer valuable insights for contemporary eco-friendly architectural design. This research investigates the sustainable design strategies of vernacular architecture in southwest Hubei, focusing on the First Granary of Xuan’en County as a representative case study. Through field investigations of indoor environments, this study explores how traditional architectural practices have addressed the region’s complex mountainous terrain and hot, humid climate. Major sustainable design strategies include rational site selection and layout adapted to the terrain, building forms and spatial organizations tailored to the environmental conditions, and the use of a "double-skin" envelope structure to enhance thermal insulation and ventilation. The results demonstrate that the average temperature of the grain depot does not exceed 25°C without active means, meeting the quasi-low temperature storage standard. Through comprehensive field research and analysis, this study demonstrates how these traditional design strategies not only improve indoor thermal comfort and energy efficiency but also align with local economic levels and modern living requirements. By leveraging passive design techniques rooted in local cultural and environmental contexts, this research provides a framework for integrating these strategies into contemporary sustainable architecture.

## Introduction

With the development of modern technology and urbanization, the number of buildings in China and worldwide has increased dramatically, and with it, the pressure on building energy consumption and environmental issues has increased. In addition, with China’s goal of "carbon peaking and carbon neutrality", the construction industry is forced to move towards a low-carbon and green sustainable development model [1]. Therefore, it is urgent to promote green buildings. Vernacular architecture, with its deep imprint of geographical environments and reflection of the relationship between humans and nature, is a testament to the adaptive strategies developed over centuries. Re-examining these traditional buildings and considering their adaptability to environmental, occupational, and living conditions can play a crucial role in reducing energy consumption while meeting building usage needs. Learning from the sustainable construction practices of traditional architecture is vital. Clearly, rethinking and thoroughly understanding the sustainable design strategies in vernacular architecture are key factors in optimizing indoor thermal environments.

Previous studies on the sustainable design of vernacular architecture have mainly focused on three aspects as shown in Table 1. Firstly, from the perspective of thermal performance of vernacular buildings, studies have been conducted on comparing the thermal performance of vernacular buildings with modern buildings. Due to the long-term regional adaptation and optimization of traditional building materials, maintenance structure construction methods, and building spatial layouts, vernacular buildings often have good thermal performance. For example, Mady Mohamed et al. [2] conducted an investigation on vernacular buildings in Asir Region of Saudi Arabia and found that traditional mud architecture have superior thermal performance over con-temporary concrete block construction. Qianqian Sun et al. [3] investigates the thermal mechanism differences between volcanic-rock dwellings and modern dwellings in Haikou, and found that the envelope of volcanic-rock dwelling has better thermal insulation performance. Secondly, studies have been conducted on energy consumption analysis of vernacular buildings. For example, Pooya Lotfabadi et al. [4] conducted a comparative study of traditional and contemporary building envelope construction techniques in terms of energy efficiency in hot and humid climates. Thirdly, research in this area focuses on summarizing sustainable design strategies and proposing contemporary transformation methods. For instance, Qian Nie et al. [5] conducted an investigation on the climate-responsive design strategies of vernacular dwellings in Khams. The aforementioned studies have approached the sustainable design of vernacular architecture from various fields and perspectives, conducting research through onsite measurements and simulations, and provided reference paths for integrating these sustainable strategies into contemporary architecture.

**Table 1:** Summary of current research on the sustainable design of vernacular architecture.

Topic	Region	Author	Building type	Results
**thermal performance of vernacular buildings**	Italy	Indrika Rajapaksha et al. [6]	Residential buildings	Internal temperatures in summer are mainly within the comfort zone; the winter temperatures are well below the comfort zone and the villas would need heating
	China	Yanan Xu et al. [7]	Residential buildings	Thermal buffering effect of the semi-outdoor alley occurs under certain outdoor air temperature, soil-adjacent ground was the heat sink of indoor space during the daytime
	Myanmar	May Zune et al. [8]	Religious buildings and other public buildings	Vernacular buildings with multistage roofs offer an opportunity to improve indoor comfort in tropical climates
**energy consumption of vernacular buildings**	Iran	Amin Mohammadi et al. [9]	Residential buildings	Context-based climatic solutions including shading, natural ventilation, and insulation of external walls and roofs achieved lower annual energy consumption
	Indonesia	Chui Ying Lee et al. [10]	Residential buildings	The use of natural building materials helps reduce the electricity demand of households in Indonesia.
	Spain	Eduardo Diz-Mellado et al. [11]	Residential buildings	The geometry of the courtyard is a key factor in the cooling energy demand of buildings.
**sustainable design strategies of vernacular buildings**	Portugal	Jorge Fernandes et al. [12]	Residential buildings	The use of glazed balconies in the North of Portugal can capture solar gains and reduce heat losses.
	Cyprus	Stavroula Thravalou et al. [13]	Residential buildings	The environmental responsiveness of sachnisi buildings in Nicosia is shaped by both climatic and functional factors, aiding passive cooling and natural ventilation.
	India	Sudhir Kumar Gupta et al. [14]	Residential buildings	Conventional vernacular houses can be more energy efficient and eco-friendly by incorporating passive cooling strategies in summer.

The southwestern region of Hubei is situated at the junction of Hunan, Hubei, and Chongqing in China. It features numerous mountains and hills, with a complex topography characterized by a stepped landscape, and is home to many ethnic minorities in China. Compared to most buildings in plain areas, buildings in Southwest Hubei must consider the complex terrain and significant local climatic conditions. Therefore, residents must build buildings that meet their needs using indigenous resources while reducing energy consumption [15]. Therefore, more and more scholars have started to study the traditional vernacular architecture of the southwest Hubei region—the stilt-ed building, which is representative of the traditional vernacular architecture of the region with excellent climate adaptability and thermal environmental stability. Cheng researched the architectural performance of traditional Tujia stilted buildings in southwestern Hubei [16]. Kui Zhao performed a detailed analysis of the architectural features of stilted buildings through a field investigation of the ancient buildings in Pengjia Village in southwest Hubei, explaining its advantages in constructing sustain-able buildings [17]. Li and Lu have studied the environmental principles encapsulated within the conventional building form with the stilted building as the main architectural form, analyzed the site selection, formal layout, and building materials, respectively, and proposed optimization strategies for the renovation of the original stilted buildings from the perspective of ecotourism [18]. Recently, Miao and Wang analyzed the advantages of traditional wood-frame buildings and modern buildings in terms of low carbon from five perspectives: material selection, transportation, construction, use, and demolition, and summarized relevant strategies from analyzing the whole life cycle of buildings [19].

Although previous researchers have studied the sustainable strategies adopted in the vernacular architecture in southwest Hubei, most studies have focused on residential buildings, while research on granaries in southwest Hubei has been relatively limited. In recent years, there has been more research on granaries in other parts of China. En Li et al.[20] investigated the historical granaries in North China Plain and found that they adopted two different strategies (temperature-first vs. humidity-first) that failed to create a desirable storage environment, thus calling for a deliberate trade-off between temperature and humidity. Yansong Wang et al.[21] investigated the granaries in the middle and lower reaches of the Fu River and found that they can maintain low temperatures and prevent moisture using ventilative stone ridges, moisture-resistant walls and heat insulation storage rooms. Jiaxin Zhang et al.[22] investigated the influences of parameters relevant to building form design on thermal performance for granary buildings in Jiangsu and Anhui, China. Due to the special needs of grain storage, buildings such as granaries have high requirements for construction techniques, including moisture proofing, drainage, heat insulation, heat preservation, and fire-fighting, which are representative of vernacular architecture [23]. By studying the climatic response mechanisms of granary buildings in the hot and humid conditions of this region, valuable insights and methods can be derived for the design of buildings with similar regulatory needs. In comparable climatic conditions, both residential and public buildings share similar requirements for thermal insulation and damp-proofing, suggesting that these sustainable strategies could have broader applications. Therefore, the investigation of vernacular granaries offers important insights into how these strategies can be adapted and optimized across various vernacular building types.

To analyze the science and practicality of low-carbon design strategies in traditional stilted buildings in the Xuan’en area to promote the thermal environment of buildings, this study conducted a three-stage analysis, including a literature review and field measurements. First, this study describes the construction environment of grain silos in the Xuan’en County area under local climatic conditions. Second, this work investigates the traditional local storage building with the First Granary of Xuan’en County as an example. The sustainable design strategies are explained from macro to micro perspectives in three aspects: planning layout, shape and form, and envelope structure. Finally, this study verifies the effectiveness of sustainable design strategies on air temperature and relative humidity by analyzing the indoor thermal environment in summer and winter. Through the analysis of granaries, a special type of building, a new perspective distinct from the previous studies on residential buildings is provided for the ecological design strategies of vernacular architecture in the southwest Hubei. By inheriting and developing local ecological construction experiences, this can serve as a reference for the sustainable design of contemporary vernacular architecture in the area.

## Research region and methods

### Study area

Xuan’en County is located in the southwest part of Hubei Province. Due to the geological structures, Xuan’en County features highly complex topography with numerous mountains scattered throughout, dividing the county into various landscapes including hills, low mountains, medium-high mountains, and high mountains [24]. Furthermore, many local ethnic minorities, including Tujia, Miao, and Dong, have gathered in the area, making it one of the representative regions concentrating on various ethnic minorities in China. Under the influence of its unique natural and social environment, the Xuan’en area has a distinctive climate environment and national culture, so it is incredible to ponder the ecological design strategy in traditional vernacular architecture in the Xuan’en area.

### Climate data

Xuan’en has a humid subtropical mountainous climate with significant monsoon influence, abundant rainfall, and high humidity throughout the year. Due to the non-zonality influence, the county’s climate forms a three-dimensional climate zone, humid year-round, with sufficient rain and heat. Fig 1 presents the monthly normal temperature over 24 hours, which ranges from 4.7°C in January to 25.9°C in July, while the yearly normal temperature is 15.7°C. The average high temperature in August can reach 31.8°C.

**Fig 1:** Temperature and precipitation of Xuan’en County.

The mountainous area above 800 meters in altitude represents more than 70% of the total area. Due to the complexity of the landscape, the climate here varies significantly with changes in altitude and topography. At the granary, 845 meters above sea level, the average annual temperature is 13.7°C, and the annual precipitation is 1,635.3 mm.

In general, the climate of Xuan’en is characterized by abundant rainfall and hu-mid and moderate conditions all year round. According to China’s National Standard of Climatic Regionalization for Architecture (GB50176-2016) [25], Xuan’en belongs to the hot summer and cold winter zone, so heat protection is an important design requirement for buildings in this climate region. The average humidity graph in Fig 2 reveals high humidity in the Xuan’en area, and ventilation is critical for buildings.

**Fig 2:** Average relative humidity of Xuan’en County.

### Test methods

#### Data acquisition

To realize and evaluate the thermal insulation performance of the First Granary of Xuan’en County in detail, it was tested at 5 points located inside and outside during two typical weather seasons, summer and winter. The test parameters of the First Granary of Xuan’en County and the external environment included air temperature and relative humidity, and no mechanical ventilation and cooling measures were used in the test area. The measurement tools include a temperature and a humidity measuring instrument, with Table 2 reporting the parameters and models of the instruments.

**Table 2:** Instrument specifications.

Test Parameter	Test Equipment	Equipment Model	Test Range	Instrument Precision
**Temperature**	AZ temperature recorder	8829	-40 ◦C~85 ◦C	±0.6 ◦C
**Humidity**	WEATHER CHECKER	8750	0%RH~100%	±3%RH
			RH	

Fig 3 illustrates the layout of the test apparatus and the measurement points. Measurement point A is at the main hall of the granary and measurement point B is at the aisle between the outer wall and the granary. It should be noted that due to the symmetry of the left and right sides of the granary, only the right side was selected for measurement. Measurement point C is located outside the granary. Measurement point D is on the outside of the outer wall corresponding to measurement point B. Measurement point E is on the inside of the outer wall of measurement point C. Additionally, to ensure the accuracy of the test, all measurements were located at 1.1m from the ground and 0.5m from the walls and obstacles, the measurement time was 12h, and the data were recorded at an interval of 1 hour.

**Fig 3:** Layout and test points of the granary.

#### Evaluation criteria

Researchers worldwide have constructed a variety of indoor thermal comfort standards regarding the indoor thermal environment, among which the ASHRAE Standard 55–2013 and the China National Standard (GB/ T50785-2012) [26, 27]. However, these standards study the indoor thermal environment of residential buildings and do not cover storage buildings. According to the Technical criterion for grain and oil-seeds storage (GB/T29890-2013) [28], grain should generally be stored in low-temperature storage, the so-called low-temperature storage, where the grain temperature is controlled year-round to be 15°C and not more than 25°C, which is called the quasi-low-temperature storage. It has been more than 70 years since the construction of the first grain depot in Xuan’en County. Considering the thermal loss of the building itself and the requirement to meet the grain storage standards, this study uses the quasi-low temperature storage standard as the benchmark, which means that the maximum local temperature does not exceed 25°C.

## Sustainable design strategy—A case study of the First Granary of Xuan’en County

### Case description

The First Granary of Xuan’en County is in Xuan’en County, Enshi Autonomous Prefecture, Hubei Province. It is one of the first grain depots built in Xuan’en County after the 1950s, providing grain storage services for six townships, including Changtanhe, Dong Township, Wanzhai Township, Zhushan Township, and Jiaoyuan Town-ship. Xuan’en County belongs to the subtropical monsoon climate zone, with four clear seasons, cold winters, and hot summers [29]. Therefore, the main building requirements for this environment are moisture-proof walls/roofs, ventilation, and heat insulation. Additionally, the First Granary of Xuan’en County is located at an altitude of 800m-1200m in the second-height mountain areas, which are humid and rainy, with insufficient light and temperature. These features are very suitable for low-temperature grain storage, and the area is less crowded, which is conducive to the safe management of the grain depot.

### Architectural layout—Adapting to the terrain

Topography and climate have been fundamental factors influencing architectural differentiation [30]. The First Granary of Xuan’en County is situated in a valley be-tween two mountains, at an elevation of approximately 845 meters (Fig 4). Located at the center of the valley wind thermal circulation, the long side of the building is arranged parallel to the mountain contour lines and perpendicular to the direction of the valley wind, effectively utilizing the valley wind to improve its ventilation conditions (Fig 5).

**Fig 4:** Grain depot storage group diagram.

**Fig 5:** Site plan of the First Granary of Xuan’en County.

### Shape and form- adapting to the climate

The First Granary of Xuan’en County is 37.6 m long and 21.7 m wide, square with an area of 788 square meters and a capacity of 800 tons. The granary adopts a simple rectangular form combined with a double-eaved hip roof, with a shape factor of 0.24, which can effectively reduce heat loss caused by the exterior surface area.

The granary in the main hall is built adopting the hanging feet technique, where 16 huge wooden columns are used as the supporting structure of the granary. Each wooden column is padded with stone piers under the granary, which is 0.56 meters high, plus the ground pillow and the bottom plate of the granary. The height of the grain storage from the ground is about 1.2 meters, forming a "stilted granary" with great local traditional architectural characteristics. The hollow bottom of the silo isolates the grain from the ground and prevents moisture from seeping up-ward. Moisture is circulated through the air duct comprising the bottom of the granary, the ground, and the wall and is then discharged through the vent set at the bottom of the outer wall, preventing rodent damage.

Natural ventilation is the main way to relieve indoor overheating in traditional buildings, which is inexpensive and does not require excessive energy consumption [31]. In summer, the prevailing wind direction in Xuan’en is from southeast. The building utilizes wind pressure to create natural ventilation: the southeast wind creates a high-pressure zone on the windward southeast gable and a low-pressure zone on the leeward northwest gable. The main entrance and windows on the southeast gable serve as air inlets, while the windows on the north gable serve as air outlets. The airflow passes through the building’s longitudinal depth, forming a cross-ventilation that carries away heat.

Additionally, the building employs a clever section design to achieve cooling through stack ventilation: the tall main hall forms a vertical shaft space, allowing indoor hot air to rise and escape through clerestory windows. Cool air enters from ventilation openings at the base of the outer walls, flows across the raised floor at the bottom of the granary, and reaches the central hall, creating stack ventilation that expels heat (Figs 6 and 7). Under the combined effects of stack and wind pressure, the granary achieves excellent ventilation, effectively regulating the indoor temperature and humidity.

**Fig 6:** Structures for ventilation. **(A)** Ventilation opening on exterior walls. **(B)** Wooden pillars and floor raised on stone pillars. **(C)** Ventilation Shaft in the Hallway. **(D)** clerestory windows.

**Fig 7:** Section of the granary showing the process of stack ventilation.

### Envelope structure- double skin

In order to alleviate the economic pressure and inaccessibility, the enclosure materials used for the First Granary of Xuan’en County are local natural materials, such as wood, marble, and clay. Wood is the main material for the granary and the roof in-side the granary, marble is the base of the granary, and clay is used for the exterior walls and roof to increase the airtightness of the enclosure. Using natural materials for the envelope can significantly reduce energy consumption while improving the stability of the thermal environment within the building [32].

Traditional buildings are often reasonably designed in terms of walls, openings, and roofs to reduce the influence of the outdoor environment on the indoor environment. Regarding the walls, normally the vernacular dwellings in Southwest Hubei only use wooden walls with cedar planks, with a thickness of about 27mm, which have limited thermal insulation performance. To improve the thermal insulation performance, the First Granary of Xuan’en County adopted different strategies. While the inner warehouse walls are made of wooden cladding as well, the outer walls are constructed with 450mm thick brick walls. These two walls are separated by a 1.5 m air gap, creating a "double-skin" cavity structure that significantly enhances the thermal insulation performance of the enclosure (Fig 8). The white lime plaster on the exterior of the brick walls also helps reduce solar heat gain.

**Fig 8:** Section of the granary.

As one of the direct sources of indoor heat, the roof substantially keeps the indoor thermal environment stable. The roof also features a "double-skin" structure, with the upper layer consisting of roof tiles and the lower part made of wooden ceiling boards. The attic space between the two serves as an air gap. The clerestory windows between the overhanging eaves facilitates ventilation and heat dissipation in the air gap.

The granary’s exterior door is made of wood, and the windows use wooden lattice designs to meet lighting needs. Additionally, there are adjustable wooden shutters in-stalled to reduce heat loss. In summer, the wooden shutters can be opened to promote the convection of hot air and lower the indoor temperature (Fig 9A). In winter, the shutters can be closed to aid in insulation (Fig 9B). Thermal parameters are shown in Table 3.

**Fig 9:** Facade of the First Granary of Xuan’en County. **(A)**Wooden shutters being open in summer to promote ventilation. **(B)** Wooden shutters closed in winter for better insulation.

**Table 3:** Thermal parameters of building envelope.

U-value of the brick wall	U-value of the wooden wall	U-value of the roof	window-wall ratio	shape factor
0.76	0.14	0.76	0.21	7.79%

## Analysis of the thermal environment

### Air temperature

Figs 10 and 11 respectively show the air temperatures inside the First Granary of Xuan’en County during summer and winter from 8:00 to 17:00 throughout the day. The order of temperature change between the 5 measurement points in summer and winter is based on point C (outdoor) > point E (outdoor) > point D (office room) > point B (aisle) > measurement point A (main hall of the granary). The temperature variation outside the silo is much larger than inside the silo, especially when the outdoor temperature rises between 11:00 and 14:00. The temperature variation inside the silo has a small variation. In summer, the thermal changes in the aisle and the main hall of the granary, which are closer to the outer wall, are similar.

**Fig 10:** Temperature change of the granary during summer.

**Fig 11:** Temperature change of the granary during winter.

Table 4 reports the temperature of each measurement point from 8:00 to 17:00 during one day in the First Granary of Xuan’en County. From the test data analysis, the average temperature inside the silo is nearly stable at 25°C, meeting the standard of quasi-low temperature storage. The average temperature outside the warehouse is much higher than 25°C, which means that the warehouse is less affected by the temperature variations outside the warehouse. The maximum temperature outside the silo during the measured period was 33.1°C, the minimum was 25.8°C, and the maximum temperature difference outside the silo was 7.3°C. The maximum temperature in the main hall of the granary was 25.9°C, and the minimum was 23.7°C during the measured period. In comparison, the maximum temperature difference between the main hall of the granary and the main hall was only 2.2°C. Hence, the temperature fluctuation in the granary’s main hall and the granary, as well as in the aisle of the granary, was smooth and much smaller than the temperature outside the granary.

**Table 4:** Data analysis of temperature in the granary.

Name	Measurement point number	Maximum	Minimum	Average	Standard deviation
**Summer**	A	25.90	23.70	24.91	0.75
	B	27.00	24.30	25.81	0.83
	C	33.10	25.80	29.53	2.07
	D	28.90	24.70	27.42	1.27
	E	31.50	25.60	29.07	1.81
**Winter**	A	12.00	8.90	10.78	0.95
	B	11.60	8.60	10.19	0.95
	C	6.90	3.80	5.43	1.03
	D	11.70	8.20	9.90	1.04
	E	7.1	3.9	5.54	1.09

Fig 11 and Table 4 highlight that the temperature variation in the granary during winter is roughly similar to that in summer, and the temperature variation outside the granary is significantly higher than inside the granary. The standard deviation of the temperature variation inside the granary is higher in summer but still much smaller than outside the granary.

### Relative humidity

Fig 12 presents the variation of relative humidity at different measurement points from 08:00 to 17:00 on a summer day. The humidity outside the silo varied greatly compared to the humidity in the main hall of the grain silo and the silo aisle, which varied very little. The humidity variation outside the silo ranged from 41.4% to 80.5%, while the humidity variation in the main hall and the aisle of the silo ranged from 74.6% to 79.5% and 71.1% to 79%. Thus, the grain silo has a nearly constant humidity state in summer.

**Fig 12:** Humidity variation of the granary during summer.

According to Fig 13 and Table 5, the humidity outside the silo ranged from 57.2% to 83% in winter. Although the temperature out-side the silo was significantly lower than inside the silo, its humidity was much higher than the average humidity of 61.13% in the main hall of the grain silo. Thus, maintaining a low humidity level in the granary helps to store the grain while maintaining a relatively low temperature. As the most important space for grain storage, the grain silo main hall provides relatively stable humidity conditions for grain storage in the summer and winter when climatic conditions fluctuate significantly.

**Fig 13:** Humidity variation of the granary during winter.

**Table 5:** Data analysis of humidity in the granary.

Name	Measurement point number	Maximum	Minimum	Average	Standard deviation
**Summer**	A	79.50	74.60	77.20	1.56
	B	79.00	71.10	74.70	2.66
	C	80.50	41.40	60.03	12.05
	D	79.5	70.5	74.48	3.05
	E	80.8	42.3	59.82	11.99
**Winter**	A	66.30	58.10	61.13	2.57
	B	72.50	66.60	69.05	1.93
	C	83.00	57.20	71.64	8.69
	D	74.2	66.9	69.85	2.24
	E	82.5	58.8	72.45	8.36

## Discussion

The First Granary of Xuan’en County is a positive response of the Xuan’en region to the complex geographical and climatic environment. One of the key factors is its low-carbon passive design. Therefore, reasonable design strategies in traditional vernacular architecture can provide a suitable indoor thermal environment and respond positively to ethnic culture, economic issues, and the natural environment. Based on field investigations and tests, the following conclusions can be drawn:

1. A reasonable architectural design strategy is the first step in stabilizing the indoor thermal environment. The granary of the grain storage bin and the outer wall are separated by a 1.5m wide aisle, which makes the environment inside the bin less affected by outside temperature and humidity changes, especially in summer, and can effectively block the heat from outside. The granary of grain storage adopts the local Tujia characteristic of "hanging foot building" technology. The bottom of the granary is nearly 1.2 meters from the ground, and the wall and the ground form a natural air duct, which takes away excess heat inside the granary through the air vent and prevents dampness. The thick walls and the raised double-layer roof absorb certain dampness in the rainy season, thus meeting the requirements of low-humidity grain storage.
2. The building envelope and building materials were selected in response to climatic and economic conditions. The exterior walls are made of clay and masonry with low thermal conductivity and a thickness of 450mm, which effectively reduces the impact of outdoor environmental changes on the interior. Additionally, windows with large openings in the direction of prevailing winds provide natural ventilation to the interior without active means, reducing energy consumption. The materials used for the base and envelope of the granary are locally sourced and are easily accessible, easily processed, and are non-polluting eco-building materials. With green buildings being strongly advocated today, the design concepts of traditional Chinese architecture, such as adapting to local conditions and taking materials from local areas, have the advantage of responding well to climate change.
3. Stilted buildings are often constructed in areas with high humidity and high-temperature environments. Through field investigations and tests, the temperature and humidity inside the grain silo vary much less than outside the silo. In summer, the standard deviations of temperature and humidity changes within 12 h in the main hall of the grain silo were 0.75 and 1.56, and those outside the silo were 2.07 and 12.05. In winter, the standard deviations of temperature and humidity changes within 12 h in the main hall of the grain silo were 0.95 and 2.57, and those outside the silo were 1.03 and 8.69. The data show that stilted grain silos can provide the right thermal environment for grain storage with reduced energy consumption.
4. Compared to the vernacular dwellings in southwestern Hubei and traditional granaries in other regions of China, the key to the successful regulation of the indoor thermal environment in the First Granary of Xuan’en County lies in the com-prehensive application and complementary advantages of spatial organization, envelope structures, traditional construction methods, and building materials. Vernacular dwellings in southwestern Hubei can achieve good ventilation and moisture resistance through means such as elevating the ground floor, but their thermal insulation performance is limited due to wooden wall’s limited insulation properties [33]. Granaries in other regions, such as the North China Plain, handle high temperature outside the granary via exploiting the envelope’s thermal resistance and thermal inertia. However, limited by the lack of scientific design, the temperature control is not effective [20]. By contrast, the First Granary of Xuan’en County improved these deficiencies by applying a double-skin enclosure structure with an air gap between the brick exterior wall and the wooden interior wall of the warehouse, greatly enhancing the thermal insulation performance. This approach continued the use of traditional materials to meet eco-nomic requirements, while the design strategies for the enclosure structure and spatial organization compensated for the poor insulation of light materials, achieving a more suitable indoor thermal environment.

However, this study has certain limitations as it remains exploratory. The article selects granaries as the vernacular architecture type that exemplifies ecological design strategies. Due to the scarcity of exsiting vernacular granaries in southwest Hubei, this study mainly focused on one well-preserved, distinctive, and representative example to explore its passive design strategies and indoor and outdoor thermal environments, and did not select more cases for a comprehensive analysis. Future research should include a larger sample size, encompassing more diverse types of vernacular buildings in southwest Hubei, to summarize their common characteristics in order to obtain more extensive and in-depth research results. Additionally, future research needs to control variables for the quantitative assessment of the effectiveness of different passive design strategies in reducing energy consumption, in order to identify and quantify the most impactful passive strategies.

## Conclusion

As a grain warehouse building using local stilted architecture techniques, the First Granary of Xuan’en County has excellent climate adaptability and can meet grain storage needs. In this study, the building design of the First Granary of Xuan’en County was analyzed, and its physical environment was monitored. The results show that following the principles of local, distinctive, and site-specific design can significantly im-prove the building’s performance. By analyzing granaries, a distinct building type, this study offers a new perspective on ecological design strategies for vernacular architecture in southwest Hubei, differing from previous residential building studies. By preserving and enhancing local ecological construction practices, and continue optimizing the sustainable design strategies, this can serve as a reference for the sustainable design of modern vernacular architecture in the region.

## Supporting information

S1 Data (XLSX)
